# Evaluation of allylestrenol for clinical pregnancies in patients treated with assisted reproductive techniques: a retrospective, propensity score matched, observational study

**DOI:** 10.1186/s12884-023-05970-2

**Published:** 2023-09-13

**Authors:** Yuexin Yu, Tingting Yu, Weiping Ding, Yinling Xiu, Mengsi Zhao, Kaixuan Sun, Qian Zhang, Xiaohang Xu

**Affiliations:** 1 Department of Reproductive Medicine, General Hospital of Northern Theater Command, Shenyang, Liaoning 110000 China; 2 Obstetrics and gynecology clinic of the 79th Army Group Hospital, Liaoyang, Liaoning 111000 China

**Keywords:** Allylestrenol, Dydrogesterone, Assisted reproductive techniques, Luteal phase support, Progesterone

## Abstract

**Background:**

Allylestrenol is an oral progestogen being increasingly used for luteal phase support in assisted reproductive techniques. However, evidence of the clinical efficacy of allylestrenol in luteal phase support is lacking. Dydrogesterone is a representative drug used for luteal phase support, the efficacy of which has been clinically confirmed. As such, we aimed to compare the effects of allylestrenol with the standard dydrogesterone on clinical pregnancy rates and pregnancy outcomes.

**Methods:**

This retrospective study included 3375 assisted reproductive technique cycles using either allylestrenol or dydrogesterone between January 2015 and March 2020. Patients using either allylestrenol or dydrogesterone were matched in a 1:1 ratio using propensity scores. The primary outcomes were clinical pregnancy rate and pregnancy outcomes.

**Results:**

No significant difference was found in the clinical pregnancy rate (53.5% *vs.* 53.2%, *P* = 0.928) and pregnancy outcomes (all *P* > 0.05) between allylestrenol and dydrogesterone. Compared with dydrogesterone, the use of allylestrenol significantly reduced the rate of biochemical pregnancies (6.4% *vs.* 11.8%, *P* < 0.001) and multiple gestation rate (16.8% *vs.* 26.3%, *P* = 0.001). Moreover, endometrial thickness, morphology, and blood flow were significantly improved by allylestrenol treatment (all *P* < 0.05).

**Conclusions:**

Allylestrenol exhibited similar effects on clinical pregnancy rates and pregnancy outcomes as dydrogesterone. Moreover, allylestrenol can significantly reduce the biochemical pregnancy rate and improve the endometrial receptivity.

## Introduction

Luteal phase support improves both implantation and pregnancy rates; thus, it is routinely administered following in vitro fertilization (IVF) or intracytoplasmic sperm injection (ICSI) to overcome luteal hormone suppression induced by controlled ovarian stimulation [1, 2]. Medication used for luteal phase support encompasses 4 main categories: progesterone, human chorionic gonadotropin (hCG), estrogen, and gonadotropin-releasing hormone analogs [3].

Progesterone therapy is the most common treatment for luteal phase support. A systematic review demonstrated that the use of progesterone was associated with a higher live birth rates and number of ongoing pregnancies and a lower risk of ovarian hyperstimulation syndrome [4]. As a natural luteal product, progesterone is a basic drug used for hormone replacement therapy. However, in clinical applications, oral progesterone has low bioavailability and is associated with adverse reactions such as sleepiness [5]. Intramuscular injection of progesterone can cause pain and local abscesses at the injection site, whereas vaginal administration of progesterone may be related to vaginal irritation, drug shedding, and bleeding [6]. Therefore, at present, other progesterone drugs are often used to reduce the dose of progesterone, especially dydrogesterone [7]. Several clinical trials have indicated that dydrogesterone is at least as efficacious as progesterone for luteal phase support [8–10], but dydrogesterone still has side effects, such as vaginal bleeding [11]. Therefore, the search for new prognostic agents with greater effectiveness and fewer side effects is ongoing.

Allylestrenol, first introduced in the 1960s, is used for recurrent miscarriage and premature labor prevention [12–14]. In China, luteal support is used off-label owing to its significant effects on progesterone receptors, serum estradiol levels, and serum progesterone levels [15]. However, little new evidence has been gathered in recent decades on whether allylestrenol can be used for luteal phase support after assisted reproductive techniques (ART) and on its effect on ART outcomes. The purpose of this study was to compare the effects of allylestrenol with dydrogesterone on ART and pregnancy outcomes and to evaluate whether allylestrenol could act as a routine luteal phase support medication in clinical practice.

## Materials and methods

### Study design and participants

This retrospective study was conducted at the Reproductive Medicine Center of the General Hospital of Northern Theater Command between January 1^st^, 2015, and March 24^th^, 2020. This study was conducted in accordance with the ethical standards and the Declaration of Helsinki. The General Hospital of Northern Theater Command Research Ethics Committee confirmed that no ethical approval was required because this was a retrospective observational study.

The study included premenopausal women > 18 or < 50 years of age who underwent IVF or ICSI with a first documented record of oocyte retrieval from the 1^st^ of January 2015 to the 24^th^ of March 2020. Women with a history of infertility for > 15 years were excluded. Other exclusion criteria included missing data on infertility duration, pregnancy outcomes, ART outcome, or abnormal endometrial morphology.

All participants received progesterone as this is the standard drug used for luteal phase support. A total of 3375 ART cycles were selected due to their extra medication, dydrogesterone, or allylestrenol. These 3375 cycles were categorized into 2 groups: dydrogesterone (2368 cycles) and allylestrenol (989 cycles).

### Data collection and outcomes

All data and outcomes were obtained from electronic medical records. Demographic data including age, type of infertility, infertility duration, baseline hormone levels (follicle-stimulating hormone, luteinizing hormone, estradiol, anti-Müllerian hormone), antral follicle count, ovarian stimulation protocol (progestin-primed ovarian stimulation, mild stimulation protocol, gonadotropin-releasing hormone antagonist protocol, modified long protocol, long protocol, luteal phase stimulation protocol), endometrial morphology, uterine blood flow, and endometrial blood flow were recorded.

The primary outcomes were ART (clinical pregnancy, non-pregnancy, and biochemical pregnancy) and clinical pregnancy outcomes (live birth, abortion, embryonic demise, and labor induction). The secondary outcomes included the number of miscarriages, ectopic pregnancy rate, and multiple pregnancy rate. Clinical pregnancy was defined as the presence of at least one intrauterine gestational sac on ultrasonography. Biochemical pregnancy was defined as a positive hCG level without gestational sac development. A live birth was confirmed by the delivery of a live neonate after 28 weeks of gestation. Abortion was defined as pregnancy loss before 28 weeks of gestation. Embryonic demise referred to the termination of embryo development before 12 weeks of gestation. Labor induction denoted the termination of pregnancy after 12 weeks of pregnancy due to maternal or fetal reasons and artificially induced uterine contraction. An ectopic pregnancy was identified as an extrauterine gestational sac on ultrasonography. Multiple pregnancies were defined as pregnancies with more than 1 fetus.

### Statistical analysis

Statistical analysis was performed using R software, version 3.3.3 (R Foundation for Statistical Computing). Categorical variables are described as the number of cases and percentages; these were compared using the chi-squared test. Continuous variables were described as median and interquartile range and analyzed using the Kruskal–Wallis test. The efficacy of therapies was assessed using univariate and multivariate analyses, and the values of odd ratio (OR) and 95% confidence interval (CI) were calculated.

Propensity score matching (PSM) was used to adjust for significant differences in the baseline characteristics of women in each group. Propensity scores were calculated using a logistic regression model. A 1:1 matching was then performed using a caliper with a width of 2. The variables included in the calculations are listed in Table 1. The standardized mean difference (SMD) was used to determine the balance of covariate distributions between groups after PSM. An SMD < 0.1 was well-balanced. A subgroup analysis stratified by the number of embryos transferred was also conducted. Statistical significance was indicated by *P* < 0.05.

**Table 1:** Patient Demographics Prior to and Post-PSM

Variables	Pre-PSM				Post-PSM			
	**Dydrogesterone** (*N* = 2,368)	**Allylestrenol** (*N* = 989)	***P*-value**	**SMD**	**Dydrogesterone** (*N* = 989)	**Allylestrenol** (*N* = 989)	***P*-value**	**SMD**
**Age (Years)**	33.00 [30.00, 36.00]	33.00 [30.00, 36.00]	0.035	0.110	33.00 [30.00, 36.00]	33.00 [30.00, 36.00]	0.396	0.052
**Type of infertility (%)**			0.189	0.051			0.368	0.043
Primary	1217 (51.4)	483 (48.8)			462 (46.7)	483 (48.8)		
Secondary	1151 (48.6)	506 (51.2)			527 (53.3)	506 (51.2)		
**Years of infertility**	4.00 [2.00, 6.00]	3.00 [2.00, 5.00]	< 0.001*	0.119	3.00 [2.00, 5.00]	3.00 [2.00, 5.00]	0.771	0.029
**Basal hormone level**								
FSH (mIU/mL)	5.88 [4.86, 7.15]	5.97 [4.89, 7.09]	0.477	0.061	5.80 [4.73, 7.10]	5.97 [4.89, 7.09]	0.062	0.063
LH (mIU/mL)	4.00 [2.70, 5.75]	3.78 [2.25, 5.52]	< 0.001*	0.109	3.86 [2.44, 5.76]	3.78 [2.25, 5.52]	0.148	0.062
E_2_ (pg/mL)	36.29 [26.38, 48.52]	34.84 [24.56, 45.86]	0.015	0.051	34.64 [25.16, 45.99]	34.84 [24.56, 45.86]	0.515	0.022
AFC	13.00 [9.00, 20.00]	14.00 [9.00, 21.00]	0.003*	0.109	14.00 [9.00, 22.00]	14.00 [9.00, 21.00]	0.607	0.029
AMH (ng/ml)	2.96 [1.74, 4.90]	2.99 [1.72, 4.77]	0.558	0.065	2.96 [1.71, 4.89]	2.99 [1.72, 4.77]	0.764	0.040
Progesterone (ng/ml)	0.45 [0.26, 0.68]	0.22 [0.13, 0.35]	< 0.001*	0.008	0.35 [0.20, 0.58]	0.22 [0.13, 0.35]	< 0.001*	0.018
**Hormone level on the day of hCG**								
FSH (mIU/mL)	12.41 [9.74, 16.09]	12.39 [9.87, 15.24]	0.264	0.112	12.07 [9.10, 15.42]	12.39 [9.87, 15.24]	0.099	0.009
E_2_ (pg/ml)	26.94 [16.50, 30.00]	30.00 [16.74, 30.00]	0.386	0.044	27.80 [16.45, 30.00]	30.00 [16.74, 30.00]	0.368	0.015
LH (mIU/mL)	1.61 [0.99, 2.65]	1.46 [0.93, 2.74]	0.065	0.017	1.38 [0.84, 2.55]	1.46 [0.93, 2.74]	0.151	0.022
AFC	12.00 [7.00, 17.00]	12.00 [8.00, 17.00]	0.068	0.060	12.00 [8.00, 18.00]	12.00 [8.00, 17.00]	0.850	0.030
Progesterone (ng/ml)	0.87 [0.58, 1.24]	0.60 [0.36, 0.97]	0.001*	0.038	0.78 [0.47, 1.18]	0.60 [0.36, 0.97]	< 0.001*	0.049
**Ovarian Stimulation Protocol (%)**			< 0.001*	0.823			0.994	0.038
PPOS	64 (2.7)	32 (3.2)			35 (3.5)	32 (3.2)		
Mild stimulation protocol	144 (6.1)	21 (2.1)			21 (2.1)	21 (2.1)		
GnRH antagonist protocol	404 (17.1)	290 (29.3)			302 (30.5)	290 (29.3)		
Modified long protocol	404 (17.1)	394 (39.8)			381 (38.5)	394 (39.8)		
Long protocol	1143 (48.3)	171 (17.3)			171 (17.3)	171 (17.3)		
Luteal phase stimulation protocol	118 (5.0)	46 (4.7)			43 (4.3)	46 (4.7)		
Others	91 (3.8)	35 (3.5)			36 (3.6)	35 (3.5)		
**Number of Miscarriages**			0.009*	0.119			0.188	0.112
0	2125 (89.7)	902 (91.2)			888 (89.8)	902 (91.2)		
1	216 (9.1)	70 (7.1)			88 (8.9)	70 (7.1)		
2	21 (0.9)	11 (1.1)			11 (1.1)	11 (1.1)		
≥ 3	6 (0.3)	2 (0.2)			2 (0.2)	2 (0.2)		

*PSM* propensity score matching, *SMD* standardized mean difference, *FSH* follicle stimulating hormone, *LH* luteinizing hormone; *E*_*2*_ estradiol, *AFC* antral follicle count, *AMH* anti- Müllerian hormone, *hCG* human chorionic gonadotropin, *PPOS* progestin-primed ovarian stimulation, *GnRH* gonadotropin-releasing hormone

^*^P < 0.05

## Results

### Baseline characteristics of participants

Between January 2015 and March 2020, 15,188 cycles of IVF or ICSI were performed at the Reproductive Medicine Center of the General Hospital of Northern Theater Command. Based on the inclusion and exclusion criteria; 8323 cycles did not meet the inclusion criteria and 340 cycles were excluded (Fig. 1). Cycles with the combined use of both dydrogesterone and allylestrenol were excluded, leaving a total of 3375 cycles included for further analysis.

**Fig. 1:** The Screening, Enrollment, and propensity score matching (PSM) of this study

The participants were well matched post-PSM in terms of baseline characteristics (Table 1). The median patient age was 33 years. A total of 1033 patients (52%) experienced secondary infertility. The median duration of infertility was 4 years. Most participants (39%) received a modified protocol for oocyte retrieval. Less than 10% of participants had miscarriages.

### Allylestrenol exhibited similar impacts on ART and pregnancy outcomes as dydrogesterone

Both the ART success rates and clinical pregnancy outcomes are shown in Table 2. Clinical pregnancies occurred in 529 of the 989 participants (53.5%) in the allylestrenol group and in 526 participants (53.2%) in the dydrogesterone group. The between-group differences were not significant. The non-pregnancy rate was 40.1% in the allylestrenol group and 35.0% in the dydrogesterone group (*P* = 0.020). Compared with dydrogesterone, the application of allylestrenol significantly reduced the rate of biochemical pregnancies (6.4% *vs.* 11.8%, *P* < 0.001) and the rate of multiple gestations (16.8% *vs.* 26.3%, *P* = 0.001). In the multivariate regression analysis, the rate of biochemical pregnancies remained significant (OR = 0.53, 95%CI = 0.389–0.705). No significant difference was found between the allylestrenol and dydrogesterone groups in terms of the clinical pregnancy rate or clinical pregnancy outcomes (Table 3).

**Table 2:** Primary and Secondary Outcomes of Allylestrenol versus Dydrogesterone after PSM

**Variables**	**Dydrogesterone** (*N* = 989)	**Allylestrenol** (*N* = 989)	***P*-value**
**ART outcomes (%)**			
Clinical pregnancy	526 (53.2)	529 (53.5)	0.928
Non-pregnancy	346 (35.0)	397 (40.1)	0.020*
Biochemical pregnancy	117 (11.8)	63 (6.4)	< 0.001*
**Pregnancy outcomes (%)**			
Live birth	422 (42.67)	416 (42.06)	0.820
Abortion	34 (3.44)	36 (3.64)	0.903
Embryonic demise	55 (5.56)	59 (5.97)	0.772
Labor induction	15 (1.52)	18 (1.82)	0.725
**Ectopic pregnancy (%)**	5 (0.5)	9 (0.9)	0.284
**Multiple gestations (%)**	111 (26.3)	70 (16.8)	0.001*

*ART* assisted reproductive techniques, *PSM* propensity score matching

^*^P < 0.05

**Table 3:** Multivariable analysis of factors associated with ART and pregnancy outcomes

Variables	Crude OR	Adjusted OR
**Clinical pregnancy**	0.89 (0.765,1.031)	0.91 (0.774,1.068)
**Biochemical pregnancy**	0.51 (0.379,0.669)	0.53 (0.389,0.705) *
**Live birth**	0.99 (0.778,1.273)	1.05 (0.810,1.358)
**Abortion**	0.78 (0.524,1.144)	0.76 (0.499,1.124)
**Embryonic demise**	1.09 (0.785,1.499)	1.03 (0.732,1.437)
**Labor induction**	1.44 (0.784,2.553)	1.42 (0.760,2.574)
**Multiple gestations**	0.56 (0.417,0.736)	0.59 (0.433,0.794)

*ART* assisted reproductive techniques, *OR* odd ratio

^*^P < 0.05

Moreover, a subgroup analysis of different numbers of transferred embryos was conducted (Table 4), and the clinical pregnancy rate, pregnancy outcomes, and multiple gestation rates were stratified by the number of embryos transferred. The rate of biochemical pregnancies was significantly lower in patients who received 1 (*P* = 0.016) or 2 embryos (*P* = 0.002). In addition, between-group differences were not remarkable in patients who received 3 embryos. Taken together, allylestrenol exhibited similar effects on ART and pregnancy outcomes as dydrogesterone, though it exerted more positive effects on biochemical pregnancies.

**Table 4:** Primary outcomes of allylestrenol versus dydrogesterone stratified by the number of embryo transferred

**Embryo(s) Transferred**	**Variables**	**Dydrogesterone** (*N* = 989)	**Allylestrenol** (*N* = 989)	***P*-value**
**1**	**Number of participants**	257	372	
	**ART outcome (%)**			
	Clinical pregnancy	124 (48.2)	205 (55.1)	0.107
	Non-pregnancy	106 (41.2)	148 (39.8)	0.776
	Biochemical pregnancy	27 (10.5)	19 (5.1)	0.016*
	**Clinical pregnancy outcomes (%)**			
	Live birth	99 (38.52)	171 (45.97)	0.076
	Abortion	8 (3.11)	10 (2.69)	0.810
	Embryonic demise	15 (5.84)	21 (5.65)	1.000
	Labor induction	2 (0.78)	3 (0.81)	1.000
	**Multiple gestations (%)**	2 (1.6)	1 (0.5)	0.658
	**Number of implantations**			0.059
	0	131 (51.0)	166 (44.6)	
	1	124 (48.2)	206 (55.4)	
	2	2 (0.8)	0 (0.0)	
	3	0(0.0)	0(0.0)	
**2**	**Number of participants**	680	602	
	**ART outcome (%)**			
	Clinical pregnancy	381 (56.0)	320 (53.2)	0.329
	Non-pregnancy	216 (31.8)	241 (40.0)	0.002*
	Biochemical pregnancy	83 (12.2)	41 (6.8)	0.002*
	**Clinical pregnancy outcomes (%)**			
	Live birth	308 (45.29)	242 (40.20)	0.075
	Abortion	22 (3.24)	26 (4.32)	0.382
	Embryonic demise	39 (5.74)	37 (6.15)	0.847
	Labor induction	12 (1.76)	15 (2.49)	0.479
	**Multiple gestations (%)**	104 (27.3)	67 (20.9)	0.062
	**Number of implantations**			0.170
	0	296 (43.5)	275 (45.7)	
	1	246 (36.2)	227 (37.7)	
	2	135 (19.9)	100 (16.6)	
	3	3 (0.4)	0 (0.0)	
**3**	**Number of participants**	52	11	
	**ART Outcome (%)**			
	Clinical pregnancy	21 (40.4)	3 (27.3)	0.637
	Non-pregnancy	24 (46.2)	5 (45.5)	1.000
	Biochemical pregnancy	7 (13.5)	3 (27.3)	0.494
	**Clinical Pregnancy Outcomes (%)**			
	Live birth	15 (28.85)	2 (18.18)	0.712
	Abortion	4 (7.69)	0 (0.0)	1.000
	Embryonic demise	1 (1.92)	1 (9.09)	0.321
	Labor induction	1 (1.92)	0 (0.0)	1.000
	**Multiple gestations (%)**	5 (23.8)	1 (33.3)	1.000
	**Number of implantations**			0.698
	0	31 (59.6)	8 (72.7)	
	1	12 (23.1)	2 (18.2)	
	2	4 (7.7)	1 (9.1)	
	3	5 (9.6)	0 (0.0)	

*ART* assisted reproductive techniques

^*^P < 0.05

### Allylestriol improved endometrial receptivity compared to dydrogesterone

Measurements of endometrial thickness, morphology, and blood flow are helpful in evaluating endometrial receptivity [16, 17]. As shown in Table 5, the proportion of endometrial type A in the allylestrenol group was higher than that in the dydrogesterone group; conversely, the proportions of endometrial type C and type B in the allylestrenol group were lower than those in the dydrogesterone group (*P* < 0.001). In terms of endometrial thickness, the left uterine artery blood flow resistance index (RI), right uterine artery blood flow RI, left uterine artery blood flow pulsatility index (PI), right uterine artery blood flow PI, peak systolic to diastolic velocity ratio (S/D) of left uterine artery blood flow, and S/D of right uterine artery blood flow were significantly higher in the allylestrenol group than those in the dydrogesterone group (*P* < 0.05). Overall, compared to dydrogesterone, allylestrenol significantly improved endometrial thickness, morphology, and blood flow, indicating a more efficient role of allylestrenol in endometrial receptivity improvement.

**Table 5:** Effects of Allylestrenol versus Dydrogesterone on Endometrial Receptivity after PSM

**Variables**	**Dydrogesterone** (*N* = 989)	**Allylestrenol** (*N* = 989)	***P*-value**
**Endometrial morphology (%)**			< 0.001*
Type A	216 (29.7)	371 (37.9)	
Type B	509 (69.9)	608 (62.1)	
Type C	3 (0.4)	0 (0.0)	
**Endometrial perfusion (%)**			0.588
I	80 (11.0)	122 (12.6)	
II	644 (88.8)	846 (87.2)	
III	1 (0.1)	2 (0.2)	
**Endometrial thickness (cm)**	0.97 (0.21)	1.00 (0.21)	0.031*
**Uterine blood flow (artery)**			
RI (left)	0.80 (0.07)	0.83 (0.34)	0.031*
RI (right)	0.80 (0.10)	0.81 (0.06)	< 0.001*
PI (left)	2.02 (0.57)	2.20 (1.39)	0.001*
PI (right)	1.96 (0.49)	2.10 (0.43)	< 0.001*
S/D (left)	5.43 (1.56)	6.03 (1.94)	< 0.001*
S/D (right)	5.32 (2.55)	5.82 (1.71)	< 0.001*
**Endometrial blood flow**			
RI	0.52 (0.11)	0.51 (0.10)	0.042*
PI	0.86 (2.02)	0.75 (0.22)	0.096
S/D	2.13 (0.56)	2.08 (0.46)	0.087

*PSM* propensity score matching, *RI* resistance index, *PI* pulsatility index; S/D: peak systolic to diastolic velocity ratio

^*^P < 0.05

## Discussion

To the best of our knowledge, this is the first study to evaluate the clinical effectiveness of allylestrenol for the treatment of luteal phase support in patients receiving ART. The results showed that allylestrenol exhibited similar effects on ART and pregnancy outcomes to dydrogesterone. The results also show that compared with dydrogesterone, allylestrenol can significantly reduce the biochemical pregnancy rate and improve the endometrial receptivity.

Luteal phase support is a common practice in ART to overcome pregnancy loss and improve implantation rate [18, 19]. Moreover, luteal phase support combined with the use of progesterone drugs, including progestogen and dydrogesterone, is routinely used in IVF/ICSI cycles. Previous studies have shown that allylestrenol is an artificially synthetic progesterone that has been used to treat abortion, intrauterine growth restriction, and threatened premature labor [20, 21]. Recently, due to the excellent bioavailability and tolerability, oral allylestrenol has been used for luteal phase support therapies. However, its efficacy in ART has never been assessed. Our results demonstrate that there was no significant difference in the clinical pregnancy rate, rate of live birth, abortion, embryonic demise, or labor induction between allylestrenol and dydrogesterone. Considering the well-established effects of dydrogesterone in ART [8, 22], we speculated that allylestrenol might be a new standard medication for luteal phase support in IVF/ICSI cycles.

Notably, the superiority of allylestrenol in decreasing the risk of biochemical pregnancies and multiple gestations was identified in this study. A total of 180 participants (9.1%) had a biochemical pregnancy, which was defined as a positive βhCG test result with no pregnancy on ultrasound. A biochemical pregnancy was confirmed in 11.8% of participants treated with dydrogesterone, and this rate was higher than the 3–5% reported in previous studies [23, 24]. This may be due to variability in ovarian stimulation protocols. The criteria for identifying patients for single embryo transfer is limited. To achieve a higher rate of ART success, multiple embryos are transferred, leading to multiple gestations [25]. In this study, the rate of multiple gestations was lower in the allylestrenol group than in the dydrogesterone group (16.8% vs 26.3%). This may be explained by the previous finding that allylestrenol could be used to avoid multiple gestations and associated complications, such as maternal morbidity, fetal and neonatal morbidity, and mortality [26].

The study also suggested a role for allylestrenol in increasing endometrial thickness and improving uterine blood flow. A thin endometrium is associated with a lower probability of conception and pregnancy complications [27]. Therefore, hormonal supplementation is routinely used for endometrial preparation for ART in patients with premature ovarian failure (POF). The endometrial thickness in the allylestrenol and dydrogesterone groups was 1 cm and 0.97 cm, respectively. This is like the endometrial characteristics of POF patients receiving dydrogesterone or estradiol [28, 29]. Thus, considering its strong effects on endometrial thickness, morphology, and blood flow, allylestrenol may also be used for treating POF. Moreover, progesterone administration can improve endometrial receptivity and the establishment and maintenance of pregnancy. However, the underlying mechanisms leading to the difference in the effects on endometrial receptivity between allylestrenol and dydrogesterone require further investigation.

The key strengths of this study include the relatively large sample size and the fact that this study is the first to compare ART and pregnancy outcomes after luteal phase support with allylestrenol and dydrogesterone. However, several limitations should be considered when considering the results. Firstly, this study was not a randomized trial and bias could not be optimally controlled, leading to potential differences that may influence the findings. However, PSM and multivariate regression were used to reduce the influence of bias. Secondly, baseline ultrasound and histology results of the endometrium and uterus were not collected. This led to a lack of time-related effects of allylestrenol on endometrial receptivity. Thirdly, safety and tolerability data were not included or analyzed.

## Conclusion

Allylestrenol exhibited similar effects on clinical pregnancy rates and pregnancy outcomes as dydrogesterone. However, allylestrenol can significantly reduce the biochemical pregnancy rate and improve the endometrial receptivity. This suggests that allylestrenol is a reasonable alternative to dydrogesterone for luteal phase support in patients receiving IVF/ICSI. Further well-designed randomized trials are required to verify these results.

## Data Availability

Because General Hospital of Northern Theater Command is a military hospital, raw data is confidential and cannot be shared. Someone wants to request the data from this study, please contact the corresponding author (Yuexin Yu, yuyuexinpingan@163.com).
